The article "Silymarin Accelerates Liver Regeneration after Partial Hepatectomy" was retracted in 2017. Reasons: duplicated images; original data or images not available; concerns about the data; concerns about the images.

# Silymarin Accelerates Liver Regeneration after Partial Hepatectomy

**DOI:** 10.1155/2015/603529

**Published:** 2015-08-03

**Authors:** Jia-Ping Wu, Chin-Chuan Tsai, Yu-Lan Yeh, Yueh-Min Lin, Chien-Chung Lin, Cecilia Hsuan Day, Chia-Yao Shen, V. Vijaya Padma, Lung-Fa Pan, Chih-Yang Huang

**Affiliations:** ^1^Graduate Institute of Basic Medical Science, China Medical University, Taichung 40402, Taiwan; ^2^School of Chinese Medicine for Post-Baccalaureate, I-Shou University, Kaohsiung 84001, Taiwan; ^3^Chinese Medicine Department, E-Da Hospital, Kaohsiung 82445, Taiwan; ^4^Department of Pathology, Changhua Christian Hospital, Changhua 50006, Taiwan; ^5^Department of Medical Technology, Jen-Teh Junior College of Medicine, Nursing and Management, Miaoli 35664, Taiwan; ^6^Orthopaedic Department, Armed Forces General Hospital, Taichung 32551, Taiwan; ^7^Department of Nursing, Meiho University, Pingtung 91202, Taiwan; ^8^Department of Biotechnology, Bharathiar University, Coimbatore 641 046, India; ^9^Cardiology Department of Taichung Armed Forces General Hospital, Taichung 32551, Taiwan; ^10^Graduate Institute of Chinese Medical Science, China Medical University, Taichung 40402, Taiwan; ^11^Department of Health and Nutrition Biotechnology, Asia University, Taichung 41354, Taiwan

## Abstract

Partial hepatectomy (PHx) is a liver regeneration physiological response induced to maintain homeostasis. Liver regeneration evolved presumably to protect wild animals from catastrophic liver loss caused by toxins or tissue injury. Silymarin (Sm) ability to stimulate liver regeneration has been an object of curiosity for many years. Silymarin has been investigated for use as an antioxidant and anticarcinogen. However, its use as a supportive treatment for liver damage is elusive. In this study, we fed silymarin (Sm, 25 mg/kg) to male Sprague-Dawley rats for 7 weeks. Surgical 2/3 PHx was then conducted on the rats at 6 hrs, 24 hrs, and 72 hrs. Western blot and RT-PCR were conducted to detect the cell cycle activities and silymarin effects on hepatic regeneration. The results showed that silymarin enhanced liver regeneration by accelerating the cell cycle in PHx liver. Silymarin led to increased G1 phase (cyclin D1/pRb), S phase (cyclin E/E2F), G2 phase (cyclin B), and M phase (cyclin A) protein and mRNA at 6 hrs, 24 hrs, and 72 hrs PHx. HGF, TGF*α*, and TGF*β*1 growth factor expressions were also enhanced. We suggest that silymarin plays a crucial role in accelerated liver regeneration after PHx.

## 1. Introduction

Liver tissue presents excellent recovery ability from surgical or toxic injury. Hepatocyte regeneration is the ability to regenerate through a compensatory growth process and then return to a nonproliferative state. We know that most liver cancer patients must receive partial liver surgical resection to protect their remaining liver function. After surgery, the hepatocytes regenerate by increasing their cell numbers. The native hepatocyte function cannot maintain the integrated whole liver function. Many hepatic liver regeneration growth drugs have been tested in partially hepatectomized (PHx) animals. Silymarin is a flavonoid complex extracted from Milk Thistle plant seeds (*Silybum marianum*). Milk Thistle seeds have been used as a medicine for centuries to treat liver diseases and they are still used today. At the turn of the 20th century, medical herbalists were using silymarin for its hepatoprotective and regeneration properties. Clinical studies have shown that silymarin (Sm) can halt and even reverse early stage liver disease in recovering alcoholics. It has also been shown to be successful in treating hepatitides B and C [1–3]. Silymarin has anti-inflammatory properties resulting from inhibiting cytokines production. Silymarin in turn increases liver regeneration and the formation of new hepatocytes. However, whether silymarin can help DNA replication and mitosis in regenerative cells is still unknown. We do know that it is absorbed in the intestine, concentrates in the bile, and probably has an enterohepatic circulation that continues to recycle through the liver [4–6]. Partial hepatectomy (PHx) triggers hepatocyte proliferation-mediated liver repair and is used widely to study the mechanisms governing liver regeneration. When injured, the liver “knows” how to accurately regulate its mass by growing and when to stop. Excessive liver mass is regulated by apoptosis. The quiescent hepatocyte regulates the disorder phenomena in the liver to maintain mass and function to protect animals in the wild from the catastrophic effects of food toxins [7–9]. There are interesting differences in the timing of cell cycle progression between partial hepatectomy and silymarin treatment after PHx. Despite being very well described, the reasons for these differences remain unclear. It is important to determine the hepatocyte replication role in liver regeneration. Based on the knowledge of liver regulation and regeneration, several growth factors are required to balance between cell cycle stimulator and inhibitor genes expressed after PHx. This may explain the liver regeneration growth process regulation [10]. We suggest that silymarin may act as a cell progression agent to induce the cell cycle progress to rebuild the lost hepatic tissue. Silymarin may enhance three available growth factors (HGF, TGF*α*, and TGF*β*1), acting as a cell cycle progression agent that triggers liver regeneration to protect the liver as a hepatoprotective agent for liver disease. HGF is a mitogenic agent for many different cell types with major effects on liver hepatic growth [11–13]. Matrix breakdown may cause a rapid release of HGF into the plasma, which occurs shortly after PHx [14]. TGF*β*1 is known to be involved in the activation of a proteolytic cascade with increased proteolysis of some hepatic biomatrix components [15]. HGF and TGF*α* may have paracrine effects on regenerating hepatocytes [16, 17]. HGF, TGF*α*, and TGF*β*1 may stimulate DNA synthesis in hepatocytes, changing the cell from proliferation or death during regeneration [18, 19]. Almost immediately, we expect major changes in the complete mitogens expression for hepatocytes and in the expression of a relatively large number of genes, after silymarin treatment [20, 21].

The article "Silymarin Accelerates Liver Regeneration after Partial Hepatectomy" was retracted in 2017. Reasons: duplicated images; original data or images not available; concerns about the data; concerns about the images.

## 2. Materials and Methods

### 2.1. Animals and Treatments

Sprague-Dawley rats were obtained from the Animal House of the National Science Council in Taiwan. The rats were housed in an environmentally controlled room, at 22 ± 5°C temperature, with relative humidity of about 60%. The animals were provided with standard food pellets and tap water. All rats were acclimatized for 1 week prior to the beginning of all experiments.

### 2.2. Preparation of Hot-Water Extract Hepatoprotective Herbal Drug, Silymarin, from Milk Thistle

The hot-water extract was prepared by boiling Milk Thistle (*Silybum marianum L.*) seed meal with distilled water for 1 hr in 100°C water. The use of hot water as an extraction solvent for Milk Thistle at temperatures above 100°C was explored. The compounds yield necessary to reach their maxima was reduced from 200 to 55(%), when the extraction temperature was increased from 100 to 140°C. The extract was filtered, freeze-dried, and kept at 4°C. The silymarin (Sm) extraction yield was 6.8 mg/g (22-23). The dried extract was dissolved in distilled water before use. Silymarin (Sm, 25 mg/kg) oral gavages at the end of the 7 weeks experiment occurred.

### 2.3. Experimental Partial Hepatectomy (PHx) and Sham Groups

Three randomly selected animals were used for each time point. After injecting ketamine subcutaneously at a dose of 30 mg/kg, liver resections consisting of 70%~85% (2/3) of the liver mass were performed in the partial hepatectomy group. Animals were anesthetized for the partial hepatectomy (PHx) using isoflurane inhalation. After 70% of hepatectomy procedure completion, the animals were administered buprenex (0.3 mg/kg in 3 mL NaCl) and then placed under a lamp to prevent hypotermy. Upon awakening, the animals were then placed into cages. The animals in the PHx and corresponding group were sacrificed at 6 hrs, 24 hrs, and 72 hrs after the operation. The animal group in which no surgery was performed was used as the control liver group and referred to as the time “0” group in the quantitated graphs. All animals were sacrificed by cervical dislocation. The remnant liver lobes were excised and washed in PBS and then immediately frozen in liquid nitrogen.

The article "Silymarin Accelerates Liver Regeneration after Partial Hepatectomy" was retracted in 2017. Reasons: duplicated images; original data or images not available; concerns about the data; concerns about the images.

### 2.4. Western Blot Analysis

Liver extracts (20 *μ*g) were run on by 12% SDS-PAGE gel for 90 min, at 100 V, and then transferred to polyvinylidene difluoride (PVDF) (Hybond-C Extra Supported, 0.45 *μ*m; Amersham, Piscataway, NJ, USA) membranes. Membranes were blocked in 5% nonfat milk (diluted in Tris-buffered saline and 0.1% Tween 20) for 30 min and probed with the appropriate primary antibody (Santa Cruz Biotechnology, Santa Cruz, CA, USA) against HGF, TGF*α*, TGF*β*1, cyclin D1, pRb, cyclin E, E2F, cyclin A, and cyclin A at 4°C overnight and then incubated with HRP-conjugated secondary antibody (Promega, Madison, WI, USA). After extensive washing, the targeted proteins were detected using an enhanced chemiluminescence system (ECL).

### 2.5. Reverse Transcriptase PCR (RT-PCR)

0.5 *μ*g of the total RNA was derived from liver plus primers using RT-PCR. The first-strand synthesis kit was applied according to the manufacturer's instructions; the PCR primers included (1) TGF*β*1: forward primer of TGF*β*1 (5′AGGAGACCATTCCCCTGACT3′); reverse primer of TGF*β*1 (5′TTCTTCCTCCACTTCCCCTT3′), (2) cyclin B: forward primer of cyclin B (5′ACCTACAGTGAAGATGCACACC3′), reverse primer of cyclin B (5′CCTGTAGTTCTTGTTTCCTGCAC3′), (3) cyclin A: forward primer of cyclin A (5′-GCAGAGTTCTGATGGAGAGA-3′), reverse primer of cyclin A (5′-ACAGTCTTGCAGGTGACATC-3′), (4) HGF: forward primer of HGF (5′-CTGCTGCAGGAGACCATGTA-3′), reverse primer of HGF (5′-CTCCGTGTGGGACAGGTAGT-3′), and (5) GAPDH: forward primer of GAPDH (5′-GGGTGTGAACCACGAGAAAT-3′), reverse primer of GAPDH (5′-CCACAGTCTTCTGAGTGGCA-3′). The RT-PCR results were analyzed based on the assessment of product sizes upon ethidium bromide-agarose gel electrophoresis. For each gene, we determined the cycle number of PCR reactions in which the PCR reaction was not saturated. The following PCR conditions were used: the initial denaturation step was conducted at 95°C, with the annealing temperature and extension at 72°C. The final extension was conducted at 72°C for 10 minutes. These conditions were applied to all reactions and the PCR products were electrophoresed on 1.2% agarose gel.

### 2.6. Immunofluorescence Analysis

Liver tissue sections were washed with 4% paraformaldehyde for 10 min and permeated using 0.01% Triton X-100, followed by blocking with 5% BSA in PBS for 30 min at room temperature. Sections were incubated with antibody Ki-67 (Santa Cruz Biotechnology, Santa Cruz, CA, USA) at room temperature for 1 hr. Following a wash in PBS, sections were incubated for 1 hr at room temperature in FITC-conjugated rabbit anti-mouse secondary antibody diluted 1 : 500 in PBS. The images were captured using a Leica DMI400B inverted Fluorescence microscope linked to camera.

The article "Silymarin Accelerates Liver Regeneration after Partial Hepatectomy" was retracted in 2017. Reasons: duplicated images; original data or images not available; concerns about the data; concerns about the images.

### 2.7. Immunohistochemistry Assay

Liver tissues were fixed in 10% buffered formalin. Fixed samples were embedded in paraffin, sectioned, and stained with hematoxylin and eosin (H&E) for histological examination. To identify cytoplasmic lipid vacuoles, 5 *μ*m thick sections were prepared from frozen tissues and incubated with BrdU. DNA synthesis was determined by counting BrdU-positive nuclei. The labeling was expressed as the total cells counted. Immunohistochemistry was performed using mouse anti-BrdU (Santa Cruz Diagnostics, Santa Cruz, CA) as antibody, using DAB stained to detect the targeted antibody expression.

### 2.8. Statistical Analysis

All data are expressed as the means ± S.E. For western blot and RT-PCR analysis, quantitation was carried out by scanning and analyzing the intensity of the hybridization signals using the FUJIFILM Imagine program. Statistical data analysis was performed using SigmaStat software. Student's *t*-test comparison was made when PHx and PHx + Sm rats are being compared against the sham group. Comparison between PHx and PHx + Sm was also made using Student's *t*-test. A *p* value of less than 0.05 and 0.01 was considered statistically significant. A two-way ANOVA was used when 24 hrs sham and 72 hrs sham rats were compared against 6 hrs sham rats and when 24 hrs PHx and 72 hrs PHx rats were compared against 6 hrs PHx rats, and comparison between 24 hrs PHx and 72 hrs PHx was made. A *p* value of less than 0.05 and 0.01 was considered to be statistically significant.

## 3. Results

During regeneration after 70% hepatectomy, the liver was divided one or two times and began to regenerate and then return to quiescence. We know that liver regeneration is a physiological response induced for maintaining homeostasis. According to Table 1, the result showed us the postoperative liver weight (g) which increased from 3.7 ± 0.67 (6 hrs PHx) to 5.3 ± 0.36 (24 hrs PHx) (*p* < 0.001 versus 6 hrs PHx), to 8.7 ± 1.71 (72 hrs PHx) (*p* < 0.0001 versus 6 hrs PHx), and to 10.8 ± 0.62 (168 hrs PHx) (*p* < 0.0001 versus 6 hrs PHx). Partial liver weight (g) at 72 hrs PHx has significantly increased but decreased at 168 hrs. In turn, the remnant liver weight (g) also decreased at 72 hrs PHx, from 4.7 ± 0.99 (at 6 hrs PHx) to 2.8 ± 0.64 (at 72 hrs PHx, *p* < 0.001 versus at 6 hrs PHx), but with no significant difference at 168 hrs. Thus, the liver regeneration (%) increased from 10.62% at 24 hrs to 76.32% at 72 hrs and from the highest to 119.55% at 168 hrs PHx. Given the above evidence, liver regeneration is time dependent. Partial hepatectomy (PHx) is a complex physiological response that takes place after the loss of hepatocytes caused by viral injury or secondary liver resection. During liver regeneration, a series of resections take place to maintain homeostasis to restore normal hepatic mass and structure. Virtually, all of the surviving hepatocytes undergo cellular proliferation due to tissue remodeling. PHx is a delayed physiological response during liver regeneration. We want to determine whether silymarin will accelerate the cell cycle to return to normal conditions during liver regeneration. Therefore, we detected cell cycle check proteins, cyclin D1/pRb in G1 phase and cyclin E/E2F in S phase, in sham, PHx, and silymarin treatment with PHx by western blot analysis. After partial hepatectomy, liver regeneration began to proliferate and cell cycle prolonged. We found G1 phase extended, from 6 hrs to 24 hrs and into S phase at 72 hrs during liver regeneration. Therefore, we could find cyclin D1 and pRb protein expression increased at 6 hrs PHx, but not significantly in cyclin E and E2F, when compared with sham, respectively (^*∗*^ *p* < 0.05 versus sham). Partial hepatectomy treatment with silymarin has strongly enhanced cyclin D1, pRb, cyclin E, and E2F protein expression levels (^*∗*^ *p* < 0.05 versus sham, ^#^ *p* < 0.05 versus PHx) (Figure 1(a)). After 24 hrs of liver regeneration, we found the strongest regeneration; cyclin D1, pRb, cyclin E, and E2F protein expression all were increased after PHx. We also could find silymarin improved this stage (^*∗*^ *p* < 0.05 versus sham, ^#^ *p* < 0.05 versus PHx) (Figure 1(b)). On the other hand, during long term 72 hrs PHx, cyclin D1, and pRb protein expression were decreased compared with sham, respectively. Silymarin also was induced (^*∗*^ *p* < 0.05 versus sham, ^##^ *p* < 0.05 versus PHx). In turn, cyclin E and E2F had increased. During this time, silymarin may has been losing functions to improve cell cycle, when compared with PHx (^##^ *p* < 0.05 versus PHx); however, compared with the sham, silymarin also increased (^*∗*^ *p* < 0.05 versus sham) (Figure 1(c)). After hepatic growth and restructuring, DNA synthesis was completed by 72 hrs and liver regeneration eventually stops. We focused on liver regeneration initiation and compared termination with it. Thus, we examined the cell cycle check point protein at different times. We examined cyclin D1/pRb in G1 phase and cyclin E/E2F in S phase protein expression by western blot analysis (Figures 2(a) and 2(b)). We found cyclin D1 was decreased at 24 hrs sham but increased at 72 hrs (^a^ *p* < 0.05 versus 6 hrs sham, ^b^ *p* < 0.05 versus 24 hrs sham). When compared with PHx at 6 hrs, 24 hrs, and 72 hrs, we found cyclin D1 at 24 hrs PHx was increased (^c^ *p* < 0.05 versus 6 hrs PHx) but at 72 hrs PHx was decreased (^c^ *p* < 0.05 versus 6 hrs PHx, ^d^ *p* < 0.05 versus 24 hrs PHx). However, pRb protein expression levels were increased only at 72 hrs sham (^a^ *p* < 0.05 versus 6 hrs sham, ^b^ *p* < 0.05 versus 24 hrs sham). However, after 24 hrs PHx, pRb protein expression was increased (^c^ *p* < 0.05 versus 6 hrs PHx). After 72 hrs PHx, pRb was decreased (^d^ *p* < 0.05 versus 24 hrs PHx). No significant difference compared with 6 hrs PHx was shown. Notwithstanding, silymarin also enhanced cyclin D1/pRb protein expression at all the three PHx times, 6 hrs, 24 hrs, and 72 hrs PHx, respectively (^*∗*^ *p* < 0.05 versus sham, ^#^ *p* < 0.05, ^##^ *p* < 0.01 versus PHx) (Figures 1 and 2(a)). On the other hand, in cell cycle S phase, we found cyclin E was increased at 24 hrs sham (^a^ *p* < 0.05 versus 6 hrs sham), but at 72 hrs sham has conversely to 6 hrs sham. After hepatectomy, we found cyclin E protein expression increased at 24 hrs PHx and more at 72 hrs PHx (^c^ *p* < 0.05, ^cc^ *p* < 0.01 versus 6 hrs PHx, ^d^ *p* < 0.05 versus 24 hrs PHx) (Figure 2(b)). On the other hand, E2F increased expression at 24 hrs and 72 hrs sham compared with 6 hrs sham (^a^ *p* < 0.05, ^aa^ *p* < 0.01 versus 6 hrs sham, ^b^ *p* < 0.05 versus 24 hrs sham). When compared with 6 hrs PHx, we found E2F protein expression increased at 24 hrs PHx but at 72 hrs PHx has more than 6 hrs and 24 hrs PHx (^c^ *p* < 0.05, ^cc^ *p* < 0.01 versus 6 hrs PHx; ^d^ *p* < 0.05, ^dd^ *p* < 0.01 versus 24 hrs PHx). However, silymarin also has strong functions to induce cyclin E/E2F protein expression after PHx (^*∗*^ *p* < 0.05 versus sham, ^#^ *p* < 0.05, versus PHx) (Figures 1 and 2(b)). Therefore, we could determine silymarin stimulated cell cycle protein expression for entry into S phase. After hepatic growth and restructuring, DNA synthesis is mostly complete by 72 hrs and liver regeneration eventually stops. We focused on liver regeneration initiation and compared termination with it. Furthermore, we detected whether silymarin regulated the cell cycle and accelerated it to become normal. We examined G2 and M phase check point protein, cyclin B and cyclin A, protein, and mRNA expression using western and RT-PCR. It is generally believed that the external controls have three important control points in the cell cycle at the end of G2 phase (G2/M transition), in mitosis, and in G1 phase. Intrinsic control mechanisms ensure that the cycle is executed completely. Therefore, we determine whether silymarin also improved the cell cycle at the end of G2 phase. We used western blot analysis and RT-PCR to detect protein and mRNA expression in the sham and PHx to determine the cell cycle. The results showed that the G2 phase check point protein, cyclin B, increased at 24 hrs and 72 hrs in the sham (^a^ *p* < 0.05 versus 6 hrs sham). However, cyclin B at 24 hrs in the PHx decreased compared with the sham at 24 and 6 hrs in the PHx, respectively. After 72 hrs in the PHx, cyclin B increased compared with the PHx at 24 hrs (^d^ *p* < 0.05, versus 24 hrs PHx) (Figure 3(a)). Cyclin B mRNA also decreased at 24 hrs in the PHx but increased at 72 hrs in the PHx (Figures 3(b) and 3(c)). Silymarin presented significant effects at 6 hrs, 24 hrs, and 72 hrs in the PHx to improve G1 phase into M phase. We also detected cyclin A protein and mRNA in the mitosis phase. We found that protein and mRNA expression increased at 24 hrs and 72 hrs in the sham. When compared with the sham, we found that cyclin A protein decreased at 6 hrs and 24 hrs in the PHx, respectively (^*∗*^ *p* < 0.05 versus sham). However, cyclin A mRNA decreased at 24 hrs in the PHx and increased at 72 hrs in the PHx, when compared with 6 hrs PHx (Figures 4(a) and 4(b)). Interestingly, during liver regeneration after PHx, we found cyclin A mRNA and protein expression increased at 72 hrs. PHx led cyclin A expression to delay to 72 hrs (Figure 4(c)). Interestingly, silymarin had no significant beneficial effect on cell cycle functions after 72 hrs PHx. To determine whether growth factors are the primary accelerated cell cycle effects, we examined liver regeneration related growth factors, HGF and TGF*α*, expression. We found that HGF protein and mRNA expression decreased at 6 hrs in the PHx, but this was not found at 72 hrs in the PHx. We also found that HGF increased after treatment with silymarin comparing the sham and PHx at 6 hrs or 72 hrs (Figures 5(a) and 5(b)). TGF*β*1 seems to be inhibited hepatocyte DNA synthesis that is negative regulator of liver growth. In order to determine whether cell proliferation and cell cycle are coordinately regulated by TGF*β*1 in regeneration, the result showed that TGF*β*1 protein was not significantly different in sham rats. However, after hepatectomy TGF*β*1 protein expression levels increased at 24 hrs PHx (^c^ *p* < 0.05 versus 6 hrs PHx), with the greatest expression at 72 hrs PHx (^cc^ *p* < 0.01 versus 6 hrs PHx, ^d^ *p* < 0.05, versus 24 hrs PHx) (Figure 6(a)). On the other hand, mRNA expression increased at 24 hrs and 72 hrs sham (Figure 6(b)). After partial hepatectomy, we also found mRNA expression increased at 24 hrs and 72 hrs PHx (^c^ *p* < 0.05, ^cc^ *p* < 0.01 versus 6 hrs PHx; ^d^ *p* < 0.05 versus 24 hrs PHx). One possibility is that TGF*β*1 is a mitoinhibitor that causes the end of regeneration. Therefore, this pointed out that liver regeneration proceeds to completion. Obviously, hepatocytes proceed through regeneration despite the TGF*β*1 increase. A further possibility is TGF*β*1 mitoinhibitory effects return by 96 hrs and hepatocyte proliferation stops between 48 and 72 hrs. Resistance to TGF*β*1 by regenerating hepatocytes may allow hepatocytes to proliferate even through TGF*β*1 concentrations increasing. Silymarin improved TGF*β*1 protein and mRNA expression (^*∗*^ *p* < 0.05, ^*∗∗*^ *p* < 0.01 versus sham; ^#^ *p* < 0.01, ^##^ *p* < 0.05 versus PHx) (Figure 6). Growth factors in the G1 phase have stronger expression. TGF*α* presented increased protein expression at 24 hrs in the PHx. This was not found at 6 and 72 hrs. After treatment with silymarin TGF*α* protein expression increased at 6 hrs, 24 hrs, and 72 hrs in the PHx. We used the Ki-67 antibody to examine immunofluorescence and Brdu antibodies using the immunohistochemistry assay to determine cell proliferation. The Ki-67 protein is present during all active phases in the cell cycle (G1, S, G2, and mitosis) but is absent from resting cells (G0). Therefore, both PHx and after PHx treatment Sm presented higher positive Ki-67 antibody expression from immunofluorescence analysis. Lower 10% was expressed as lower proliferation. PHx is a hyperplasia considered to be a physiological response to a specific stimulus. PHx and Sm-treated cells with hyperplastic growth remained subject to normal regulatory control mechanisms (Figure 7(a)) (green color). And Ki-67 staining is different and BrdU staining is detected only in the S phase of the cell, which is in the DNA replication phase of the cell. BrdU is a uridine derivative that will replace thymidine incorporated into the DNA of cells in S phase (Figure 7(b), yellow arrows). Brown color BrsU nuclear cells were observed at 24 hrs and 72 hrs PHx and Sm-treated cells. We suggest that silymarin could lead cell cycle accelerated and made delated cell cycle run fastly to feedback normal (Figure 8). During 72 hrs PHx, silymarin may deliver in the aggregate a set of signals that lead to regeneration termination in the cyclin A phase. Silymarin can function as a hepatoprotectant agent. In the future, silymarin may be useful as an adjuvant for the treatment of specific liver diseases.

The article "Silymarin Accelerates Liver Regeneration after Partial Hepatectomy" was retracted in 2017. Reasons: duplicated images; original data or images not available; concerns about the data; concerns about the images.

## 4. Discussion

Silymarin, a flavonoid complex extracted from Milk Thistle seeds, has been used for centuries to treat liver diseases and it is still used today as an important contributor to the support of healthy liver function [22, 23]. The liver is one of the most complex organs, playing an important role in digestion, detoxification, blood sugar regulation, and fat metabolism. Liver regeneration induced by surgical injury is an orchestrated response [24–26]. Silymarin is currently the world's most effective treatment for liver disease. It has shown positive effects in treating nearly every known form of liver disease including cirrhosis, hepatitis, necrosis, and liver damage due to drug and alcohol abuse. Many medical studies have shown that liver damage from alcohol, drugs, pesticides, some poisons, and hepatitis can be prevented or repaired with silymarin extract. In order to set in the optimal mass in relationship to its body size, the liver induces compensatory hyperplasia mechanisms. The herbal medicine, silymarin, has been used to treat liver disorders for thousands of years in the East. Silymarin has shown positive effects in treating nearly every known form of liver disease. The prognosis for a patient with a hepatic tumor after surgery is improved with silymarin treatment. The sooner the tumor growth is caught depending on the size and type, the more likely the patient will survive. Partial hepatectomy (PHx) has now become a promising therapy internationally for pathological liver conditions [27]. After hepatectomy, silymarin induces cellular proliferation and inhibits apoptosis resulting in tissue remodeling and restoration to normal hepatic mass [28, 29]. Our previous report reveals that silymarin effectively cyclin D1 and E1 thereby potentially induce cellular proliferation. However, their effect on other cyclins and on how the improvement in cellular proliferation translates into effective hepatic health is not known yet. This study investigated the silymarin action mechanisms that improve cell cycle machinery regulation after partial hepatectomy (PHx). Similar to our previous findings, silymarin enhanced cyclin D1 and cyclin E1. Further, the results show that silymarin upregulated cyclin A and cyclin B at various time intervals. Following hepatectomy, liver regeneration triggers postponed cell cycle. We determined that PHx delayed cell cycle comprised at least 2 critical phases: (a) the transition of the quiescent hepatocytes into G1 phase [30, 31], (b) the transition of the restriction point in the G1 to S phase of the cycle [32–34]. We found that, from 6 hrs to 24 hrs, the liver remains in the G1 phase, until 72 hrs liver regeneration into S phase; however, one cell cycle run presumably 24 hrs. In other words, 3 cycles are run within 72 hrs. Recent accumulating evidence indicates that silymarin may act as a cell cycle progression agent to trigger regeneration after PHx from G1 phase into S phase (Figures 1 and 2). Silymarin (Sm) has the ability to influence partial hepatectomy programmed cell cycle. Overall, silymarin induced the strongest effects at 24 hrs; however, an oral dose achieved in experimentation half-life is approximately at 72 hrs. Furthermore, we found silymarin induced them at stopped for long-term 72 hr PHx. Protein synthesis is also stimulated, thereby accelerating the regeneration process and the production of liver cells. Efficacy in the restoration of liver function and liver regeneration has been established. Our previous report highlights the potential of silymarin to enhance the growth factors such as the HGF at various time points [35]. Similarly, it should be noted, from the present study, that HGF as well as other growth factors such as TGF*α* and TGF*β*1 is also stimulated by silymarin after PHx in a similar fashion. Silymarin is a protective drug for several liver diseases. It presents only minor side effects and a good safety profile and most importantly is affordable for patients. The results from this study suggest that silymarin has considerable therapeutic potential, protecting intact liver cells, or cells not yet irreversibly damaged, by acting on the cell membranes to prevent the entry of toxic substances (Figure 7). Silymarin was recently reported to present the best liver regeneration effects. A toxicity study on silymarin observed that the seed extract is nontoxic and caused no death up to a dose of 3.2 g/kg orally. It is safe and was used in doses for further studies. The whole silymarin plant is rich in novel anticarcinogen substances and sesquiterpene lactones [36]. The present study addresses an area of special interest, liver regeneration treatment after partial hepatectomy. All of the liver cells proliferate to rebuild the lost hepatic tissue. The initiation of synthesis occurs in hepatocytes after surgery. Silymarin accelerates the cell cycle in the G1 to S phases.

The article "Silymarin Accelerates Liver Regeneration after Partial Hepatectomy" was retracted in 2017. Reasons: duplicated images; original data or images not available; concerns about the data; concerns about the images.

## Figures and Tables

**Figure 1:** Silymarin accelerates cell cycle from G1 phase to S phase during liver regeneration. Expression protein levels for G1 and S phase checkpoint proteins, cyclin D1, pRb, cyclin E, and E2F in Sham, PHx, and silymarin (Sm) treatment PHx by western blot. (a) At 6 hrs PHx, (b) at 24 hrs PHx, and (c) at 72 hrs PHx. Quantification of densitometry analysis of protein expression levels. All data are presented as means ± SEM,  ^*∗*^ *p* < 0.05, ^*∗∗*^ *p* < 0.01, as compared with the corresponding sham group.  ^#^ *p* < 0.05, ^##^ *p* < 0.01, as compared with the corresponding PHx. *α*-Tubulin was used as a loading control for western blotting.

**Figure 2:** Partial hepatectomy is a delayed cell cycle physiological response. (a) Quantification of western blot densitometry analysis of G1 phase checkpoint proteins, cyclin D1 and pRb, expression levels in Sham, PHx, and silymarin (Sm) treatment partial hepatectomy at 6 hrs, 24 hrs, and 72 hrs. All data are presented as means ± SEM, ^*∗*^ *p* < 0.05, as compared with the corresponding sham group. ^#^ *p* < 0.05, ^##^ *p* < 0.01, as compared with the corresponding PHx. ^a^ *p* < 0.05 as compared with 6 hrs sham group. ^b^ *p* < 0.05 as compared with 24 hrs sham group. ^c^ *p* < 0.05 as compared with 6 hrs PHx group. ^d^ *p* < 0.05 as compared with 24 hrs PHx group. (b) Quantification of western blot densitometry analysis of S phase checkpoint proteins, cyclin E and E2F, expression levels in Sham, PHx, and silymarin (Sm) treatment partial hepatectomy at 6 hrs, 24 hrs, and 72 hrs. All data are presented as means ± SEM; ^*∗*^ *p* < 0.05, ^*∗∗*^ *p* < 0.01 as compared with the corresponding sham group. ^#^ *p* < 0.05, as compared with the corresponding PHx. ^a^ *p* < 0.05, ^aa^ *p* < 0.01 as compared with 6 hrs sham group. ^b^ *p* < 0.05 as compared with 24 hrs sham group. ^c^ *p* < 0.05, ^cc^ *p* < 0.01, as compared with 6 hrs PHx group. ^d^ *p* < 0.05, ^dd^ *p* < 0.01 as compared with 24 hrs PHx group. (c) Representative cell cycle in sham and PHx at 6 hrs, 24 hrs, and 72 hrs three different times.

**Figure 3:** Silymarin accelerates liver regeneration after partial hepatectomy in rats by a mechanism related to G2 phase in cell cycle. (a) Expression protein levels of G2 phase checkpoint protein, cyclin B, were increased in treatment Sm after 6, 24, and 72 hrs of partial hepatectomy (PHx). Quantification of densitometry analysis of protein expression levels. All data are presented as means ± SEM, ^*∗*^ *p* < 0.05, as compared with the corresponding sham group. ^#^ *p* < 0.05 as compared with the corresponding PHx. ^a^ *p* < 0.05 as compared with 6 hrs sham group. ^c^ *p* < 0.05 as compared with 6 hrs PHx group. ^d^ *p* < 0.05 as compared with 24 hrs PHx group. *α*-Tubulin was used as a load control for western blotting. (b) Reverse transcriptase-polymerase chain reaction (RT-PCR) analysis of cyclin B mRNA expression that was increased in treatment Sm after 6, 24, and 72 h PHx. Quantification of densitometry analysis of mRNA expression levels. All data are presented as means ± SEM, ^*∗*^ *p* < 0.05, as compared with the corresponding sham group. ^#^ *p* < 0.05 as compared with the corresponding PHx. ^c^ *p* < 0.05 as compared with 6 hrs PHx group. ^d^ *p* < 0.05 as compared with 24 hrs PHx group. GAPDH was used as a load control for RT-PCR. (c) Representative cell cycle in sham and PHx at various times.

The article "Silymarin Accelerates Liver Regeneration after Partial Hepatectomy" was retracted in 2017. Reasons: duplicated images; original data or images not available; concerns about the data; concerns about the images.

**Figure 4:** Hepatic expression of cell cycle progression associated with silymarin (Sm) in liver regeneration by western blot and RT-PCR analysis. (a) Silymarin cannot hold cell cycle life in rat liver regeneration after partial hepatectomy in 72 hrs. Equal amounts of proteins lysate were separated by 12.5% SDS-PAGE by western blotting with antibodies to cyclin A. *α*-Tubulin was used as a load control for western blotting. Quantification of densitometry analysis of protein expression levels. All data are presented as means ± SEM, ^*∗*^ *p* < 0.05, as compared with the corresponding sham group. ^#^ *p* < 0.05, ^##^ *p* < 0.01 as compared with the corresponding PHx. ^a^ *p* < 0.05, ^aa^ *p* < 0.01 as compared with 6 hrs sham group. ^b^ *p* < 0.05 as compared with 24 hrs sham group. ^c^ *p* < 0.05, ^cc^ *p* < 0.01 as compared with 6 hrs PHx group. ^d^ *p* < 0.05, ^dd^ *p* < 0.01 as compared with 24 hrs PHx group. (b) RT-PCR cyclin A mRNA expression analysis showed decrease after silymarin treatment after PHx at 24 hrs and 72 hrs. GAPDH was used as a load control for RT-PCR. Quantification of densitometry analysis of mRNA levels. All data are presented as means ± SEM, ^*∗*^ *p* < 0.05, as compared with the corresponding sham group. ^#^ *p* < 0.05, as compared with the corresponding PHx. ^a^ *p* < 0.05 as compared with 6 hrs sham group. ^c^ *p* < 0.05 as compared with 6 hrs PHx group. ^d^ *p* < 0.05 as compared with 24 hrs PHx group.

**Figure 5:** The effect of silymarin (Sm) on hepatocyte proliferation after PHx. (a) Silymarin (Sm) induced HGF protein and mRNA expression at 6 hrs PHx using western blot and RT-PCR analysis. Densitometry analysis quantification of protein and mRNA expression levels; all data are presented as mean ± SEM, ^**∗**^ *p* < 0.05 as compared with the corresponding sham group. ^#^ *p* < 0.05, as compared with the corresponding PHx. *α*-Tubulin was used as a loading control for western blotting. GAPDH was used as a load control for RT-PCR. (b) Silymarin (Sm) induced HGF protein and mRNA expression at 72 hrs PHx using western blot and RT-PCR analysis. Quantification of densitometry analysis of protein and mRNA expression levels; all data are presented as mean ± SEM, ^**∗**^ *p* < 0.05, as compared with the corresponding sham group. ^#^ *p* < 0.05 as compared with the corresponding PHx. *α*-Tubulin was used as a load control for western blotting. GAPDH was used as a loading control for RT-PCR. (c) Silymarin (Sm) induced TGF*α* protein expression from 6 to 72 h PHx by western blot.

The article "Silymarin Accelerates Liver Regeneration after Partial Hepatectomy" was retracted in 2017. Reasons: duplicated images; original data or images not available; concerns about the data; concerns about the images.

**Figure 6:** TGF*β*1 contributed in some way to the events leading hepatocytes from the G0 phase to the G1 phase of the cell cycle in liver regeneration after partial hepatectomy. (a) Equal amounts of protein lysates were separated by 12% SDS-PAGE by western blotting with antibodies to TGF*β*1. Protein expression levels were increased in treatment silymarin (Sm) after 6 hrs, 24 hrs, and 72 hrs PHx. Quantification of densitometry analysis of protein expression levels. All data are presented as means ± SEM, ^*∗*^ *p* < 0.05, ^*∗∗*^ *p* < 0.01, as compared with the corresponding sham group.   ^#^ *p* < 0.05 as compared with the corresponding PHx. ^c^ *p* < 0.05, ^cc^ *p* < 0.01 as compared with 6 hrs PHx group. ^d^ *p* < 0.05 as compared with 24 hrs PHx group. *α*-Tubulin was used as a load control for western blotting. (b) RT-PCR analysis of TGF*β*1 mRNA expression during liver regeneration. Quantification of densitometry analysis of mRNA expression levels. All data are presented as means ± SEM, ^*∗*^ *p* < 0.05, as compared with the corresponding sham group.   ^#^ *p* < 0.05 as compared with the corresponding PHx. ^a^ *p* < 0.05, ^aa^ *p* < 0.01 as compared with 6 hrs sham group. ^b^ *p* < 0.05 as compared with 24 hrs sham group. ^c^ *p* < 0.05, ^cc^ *p* < 0.01 as compared with 6 hrs PHx group. ^d^ *p* < 0.05 as compared with 24 hrs PHx group. GAPDH was used as a loading control for RT-PCR.

**Figure 7:** Silymarin accelerates cell cycle from G1 phase to S phase during liver regeneration. (a) Immunofluorescence analysis of Ki-67 antibody after PHx at 6 hrs, 24 hrs, and 72 hrs and presence of silymarin treatment at 6 hrs, 24 hrs, and 72 hrs. Green points express Ki-67 stained hepatocytes. (b) Immunohistochemical staining of BrdU after PHx at 6 hrs, 24 hrs, and 72 hrs and presence of silymarin treatment at 6 hrs, 24 hrs, and 72 hrs. Yellow arrows point to positively BrdU stained hepatocytes nuclei.

**Figure 8:** Silymarin improves liver regeneration. Silymarin accelerated cell cycle in liver regeneration after partial hepatectomy (PHx). Growth factors, HGF, TGF*α*, and TGF*β*1, leading to the cell cycle running fast after silymarin treatment during liver regeneration. Silymarin makes the prolonged PHx cell cycle become normal. G1 phase check point protein: cyclin D1 and pRb. S phase check point protein: cyclin E and E2F. G2 phase check point protein: cyclin B, and M phase check point protein: cyclin A.

**Table 1:** Liver regeneration after PHx.

	6 hrs	24 hrs	72 hrs	168 hrs
Animal number (*N*)	6	6	8	10
Body weight (g)	236.7 ± 23.59	259.2 ± 10.68	234.4 ± 19.16	216.7 ± 11.25
*p* value versus 6 hrs		*p* = 0.059	*p* = 0.844	*p* = 0.0314
Postoperative liver weight (g)	3.7 ± 0.67	5.3 ± 0.36	8.7 ± 1.71	10.8 ± 0.62
*p* value versus 6 hrs		*p* < 0.001	*p* < 0.0001	*p* < 0.0001
Partial liver weight (g)	6.2 ± 0.94	6.9 ± 0.45	7.7 ± 0.63	5.8 ± 0.60
*p* value versus 6 hrs		*p* = 0.086	*p* = 0.004	*p* = 0.309
Remnant liver weight (g)	4.7 ± 0.99	4.7 ± 0.46	2.8 ± 0.64	3.9 ± 0.47
*p* value versus 6 hrs		*p* = 0.934	*p* = 0.001	*p* = 0.058
Liver regeneration (%)	−19.2	10.62	76.32	119.55

The article "Silymarin Accelerates Liver Regeneration after Partial Hepatectomy" was retracted in 2017. Reasons: duplicated images; original data or images not available; concerns about the data; concerns about the images.

## Abbreviations

HGF: Hepatocyte growth factor
PHx: Partially hepatectomized
Sm: Silymarin
ERK: Extracellular signal-regulated kinase.
